# Classification of Alzheimer's Disease and Mild Cognitive Impairment Based on Cortical and Subcortical Features from MRI T1 Brain Images Utilizing Four Different Types of Datasets

**DOI:** 10.1155/2020/3743171

**Published:** 2020-09-01

**Authors:** Saidjalol Toshkhujaev, Kun Ho Lee, Kyu Yeong Choi, Jang Jae Lee, Goo-Rak Kwon, Yubraj Gupta, Ramesh Kumar Lama

**Affiliations:** ^1^School of Information Communication Engineering, Chosun University, 309 Pilmun-Daero, Dong-Gu, Gwangju 61452, Republic of Korea; ^2^National Research Center for Dementia, Chosun University, 309 Pilmun‐Daero, Dong‐Gu, Gwangju 61452, Republic of Korea; ^3^Department of Biomedical Science, College of Natural Sciences, Chosun University, 309 Pilmun‐Daero, Dong‐Gu, Gwangju 61452, Republic of Korea

## Abstract

Alzheimer's disease (AD) is one of the most common neurodegenerative illnesses (dementia) among the elderly. Recently, researchers have developed a new method for the instinctive analysis of AD based on machine learning and its subfield, deep learning. Recent state-of-the-art techniques consider multimodal diagnosis, which has been shown to achieve high accuracy compared to a unimodal prognosis. Furthermore, many studies have used structural magnetic resonance imaging (MRI) to measure brain volumes and the volume of subregions, as well as to search for diffuse changes in white/gray matter in the brain. In this study, T1-weighted structural MRI was used for the early classification of AD. MRI results in high-intensity visible features, making preprocessing and segmentation easy. To use this image modality, we acquired four types of datasets from each dataset's server. In this work, we downloaded 326 subjects from the National Research Center for Dementia homepage, 123 subjects from the Alzheimer's Disease Neuroimaging Initiative (ADNI) homepage, 121 subjects from the Alzheimer's Disease Repository Without Borders homepage, and 131 subjects from the National Alzheimer's Coordinating Center homepage. In our experiment, we used the multiatlas label propagation with expectation–maximization-based refinement segmentation method. We segmented the images into 138 anatomical morphometry images (in which 40 features belonged to subcortical volumes and the remaining 98 features belonged to cortical thickness). The entire dataset was split into a 70 : 30 (training and testing) ratio before classifying the data. A principal component analysis was used for dimensionality reduction. Then, the support vector machine radial basis function classifier was used for classification between two groups—AD versus health control (HC) and early mild cognitive impairment (MCI) (EMCI) versus late MCI (LMCI). The proposed method performed very well for all four types of dataset. For instance, for the AD versus HC group, the classifier achieved an area under curve (AUC) of more than 89% for each dataset. For the EMCI versus LMCI group, the classifier achieved an AUC of more than 80% for every dataset. Moreover, we also calculated Cohen kappa and Jaccard index statistical values for all datasets to evaluate the classification reliability. Finally, we compared our results with those of recently published state-of-the-art methods.

## 1. Introduction

The occurrence of the most serious and common neurodegenerative disease, Alzheimer's disease (AD), is dramatically increasing among the elderly. Among people of ages ranging from 60 to 84, 24.3 million are suffering from AD [1]. The early diagnosis of AD and the best prognosis of mild impairment are possible because of an increasing list of possible biomarkers (from genetics, cognition, proteomics, and neuroimaging) [2]. Mild cognitive impairment (MCI) is the level between the predictable cognitive deterioration of regular aging and the more serious decline of dementia. At the beginning of the MCI stage, there might be difficulties with thinking, language, and memory that are more than ordinary age-related changes. A reason for differentiating the above patients from those with prodromal AD at the MCI level is that intervention early in the course of the illness may help postpone the onset and reduce the risk of AD [3]. Such intervention later in the progression of the illness might limit the disease, but it might not be possible to shift the pathology-induced neurological damage after it has already occurred. Therefore, analysis and identification of presymptomatic AD at the MCI point are highly important. Such treatment will be much more central and compelling as improved treatment becomes available.

In neuroimaging, the main task is labeling anatomical structures in magnetic resonance imaging (MRI) brain scans with accuracy. For clinical decision-making, regional volume measurement is important, as well as accurate segmentation [4]. Currently, there is no treatment method for AD, but many drugs are under development, and it is predicted that a cure will be found soon. Therefore, neuroimaging makes an optimistic prognosis more likely, and assessments by structural MRI (sMRI) can be used to check medial temporal lobe (MTL) and positron emission tomography (PET) fluorodeoxyglucose (FDG) or amyloid results. Medial temporal lobe frameworks are essential for producing new memories and for the improvement of AD [5]. Medial temporal lobe atrophy (MTA) degeneration and the associated episodic memory impairment are label features of AD, and both impair over the method of illness [5, 6]. Moreover, MTA is determined by utilizing region of interest- (ROI-) based [7], voxel-based [8], and vertex-based [5] approaches. In this research, the focus is on binary arrangement among AD, health control (HC), early MCI (EMCI), and late MCI (LMCI) utilizing sMRI. According to the atrophy assessment from MRI scans, the level of neurodegeneration and intensity can be determined. Studies have used morphometric approaches, such as the volume of interest (VOI) and ROI voxels for automatic segmentation of sMRI images. The sMRI volume involves measurement of the medial progressive lobe and hippocampus [9]. Numerous machine-learning methods have been implemented to differentiate the binary classifications of AD, HC, and MCI due to AD (mAD) and asymptomatic AD (aAD). Only using unique modalities, such as the hippocampus or amyloid imaging biomarkers, could be less sensitive in analyzing AD progression, mostly at the symptomatic level. Currently, the relevance of biomarkers for neurodegeneration, which is an analytical component of AD pathophysiology in prodromal and early-stage dementia, is widely acknowledged [10]. The most-important biomarkers for early detection of AD are the volumetric measurement of cortical thickness and subcortical volume. Studying the cortical thickness is an extensively recognized method for investigating the size of gray matter atrophy and is at the cutting edge of AD research. Cortical thinning has been found in MCI and AD [11]. However, for subcortical neurofibrillary tangle and amyloid construction in AD, MRI investigation has recently drawn attention to AD-correlated subcortical complex changes. New segmentation methods can assess subcortical volumes and provide a basis for subcortical shape analysis [11]. Many classification algorithms and approaches are based on machine learning, such as support vector machine (SVM), *k*-nearest neighbor (KNN), random forest (RF), and other ensemble classifiers. Among these, the SVM algorithm is commonly utilized because of its good accuracy and sensitivity that can deal with high-dimensional data. The SVM classification method provides a first step for recognizing data from the training dataset included in well-characterized subjects with known states, for which labels are given for the subjects [12]. The margin of the training data is maximized by composing the optimal splitting hyperplane or regular hyperplanes in a solitary or higher-dimensional plane with proposed classifier. At the testing stage, a test dataset is based on the hyperplane learned in the classification [13]. It is common for T1-weighted MRI images of each subject to be separated automatically into ROIs according to three anatomical views (sagittal, coronal, and axial), as shown in Figure 1. They are used as features for classification.

Recently, Liu et al. [14] proposed deep learning based on multiclass classification among normal control (NC), MCI not converted (ncMCI), MCI transformers converted (cMCI), and AD patients grounded on 83 ROI of MRI images and the conforming disclosed PET images. Stacked autoencoders were utilized as unsupervised learning to gain high-level features, and softmax logistic regression was adopted as a classifier. Nozadi et al. [15] researched an approach for a pipeline utilizing learned features from semantically labeled PET images to show group classification. In that research, the ADNI dataset was used, and the results were validated. In classification, they used SVM classifier with radical basis function (RBF) kernel and random forest (RF) with FDG and AV-45 biomarkers of PET image modality for AD, NC, EMCI, and LMCI groups. The FDG-PET shows good accuracy such as 91.7% for AD versus NC with RBF-SVM classifier compared to AV-45-PET. Moreover, FDG-PET demonstrates better results for EMCI versus LMCI with RBF-SVM than AV-45-PET. Gupta et al. [16] proposed a machine-learning-based framework to distinguish subjects with AD from those with MCI by using four different biomarkers: sMRI, the apolipoprotein E (APOE) genotype, cerebrospinal fluid (CSF) protein level, and FDG-PET from the ADNI dataset. According to binary classification, the combined method showed area under the receiver operating characteristic curves of 98.33%, 93.59%, 96.83%, 94.64%, 96.43, and 95.24% for AD versus HC, MCI stable (MCIs) versus cMCI, AD versus MCIs, AD versus cMCI, HC versus cMCI, and HC versus MCIs, respectively. Gorji and Naima [17] have employed a convolutional neural network (CNN) based deep learning approach for discriminating healthy people from patients with EMCI and LMCI. In their research, the ADNI dataset was used, and their proposed method has gained 94.54% accuracy, 91.70% sensitivity, and 97.96% specificity with the sagittal part of MRI for CN versus LMCI. Chyzhyk et al. [18] utilized lattice-independent component analysis to combine the kernel transformation of data with the feature section stage. The generalization of the dendritic computing classifiers was developed by that approach. For classification of NC versus AD patients, they also used the OASIS dataset and method with an accuracy of 74.75%, sensitivity of 96%, and specificity of 52.5%. Zang et al. [19] utilized operative feature consequent from functional brain network of three frequency bands during resting states for the efficiency of the classification context to classify subjects with EMCI versus LMCI. Their approached method demonstrates that the functional network features chosen by the minimal redundancy maximal relevance (mRMR) algorithm improve the distinguishing between EMCI versus LMCI compared with others chosen by stationary selection (SS-LR) and Fisher score (FS) algorithms. The chosen slow-5 band shows better accuracy compared with other bands such as 83.87% accuracy, 86.21% sensitivity, and 81.21% specification for EMCI versus LMCI. Cuingnet et al. [20] employed 10 approaches for clinically abnormal subject versus healthy groups by using an sMRI-based feature extraction technique. This approach included three methods based on cortical thickness, and five voxel-based and two other methods for the hippocampus. When the technique was used, AD versus HC achieved 81% sensitivity and 95% specificity; stable MCI and progressive MCI (P-MCI) had a sensitivity of 70% and specificity of 61%; and HC versus P-MCI had 73% and 85% sensitivity and specificity, respectively. Farhan et al. [21] utilized the right and left areas of the hippocampus, as well as the volume of gray matter, white matter, and CSF extracted from sMRI brain images. Then, four types of classification were evaluated to achieve good accuracy: SVM, multilayer perceptron, j48, and an ensemble classifier. The ensemble classifier had a high accuracy of 93.75%. Cho et al. [22] studied the incremental learning process based on the longitudinal frequency, which is represented by cortical thickness implemented on 131 ncMCI and 72 cMCI subjects. When the method was used for cMCI versus ncMCI, the sensitivity and specificity were 63% and 76%, respectively, which is a better result than that reported previously [21]. Wolz et al. [23] employed four kinds of automatic feature extraction methods (manifold-based learning, cortical thickness, tensor-based morphometry, and hippocampal volume) based on sMRI for 834 subjects from the ADNI dataset AD versus MCI and AD versus HC groups. The linear discriminant analysis (LDA) and SVM classification techniques were compared by manipulating MCI prediction and AD classification. In AD versus HC classification, LDA achieved 89% accuracy, and the sensitivity and specificity were 93% and 85%, respectively. Specifically, fusion features and the LDA classifier showed the best result for the classification of MCI-converted and MCI-stable subjects (68% accuracy, 67% sensitivity, and 69% specification). Recently, Gupta et al. [5] proposed four classifier methods—SVM, *k*-nearest neighbors, softmax, and naïve Bayes (NB)—for binary classification of AD versus HC, HC versus mAD, and mAD versus aAD and for tertiary classification of AD versus HC versus mAD and AD versus HC versus aAD utilizing subcortical and cortical features based on 326 subjects downloaded from the Gwangju Alzheimer's disease and Related Dementia (GARD) dataset website. The segmented dataset was parceled into a 70 : 30 ratio, and 70% was used as a training set. The remainder was used to obtain unbiased estimation performance as a test set. PCA was manipulated for dimensionality reduction purposes and obtained a 99.06% F1 score by the softmax classifier for AD versus HC binary classification. The SVM classifier achieved for HC versus mAD, AD versus aAD binary, and AD versus HC versus mAD tertiary classification F1 scores of 99.51%, 97.5%, and 99.99%, respectively. NB performed well for AD versus HC versus aAD tertiary classification with an F1 score of 95.88%. Moreover, to confirm the efficiency of the model, the OASIS dataset was employed.

Compared to related early works, this research addresses improving the accuracy and constancy of binary classification by comparing it with three kinds of geographical sMRI dataset. Moreover, all related works used different types of automated feature extraction method and segmentation toolbox. This work focused on the best accurate and clear segmentation method, which is multiatlas label propagation (MALP) with expectation–maximization- (EM-) based refinement (MALPEM) [24]. The best classifier, RBF-SVM, was utilized with the proposed classifier method. The GARD dataset was employed to classify the AD versus NC and EMCI versus LMCI binary classifications based on subcortical volume and cortical thickness from the sMRI brain images. Finally, the segmented features were passed through the RBF-SVM classifier and compared to the other three sMRI datasets.

## 2. Materials and Methods

### 2.1. Subjects

The data used in this study were collected from the NRCD, National Alzheimer's Coordinating Center (NACC), Alzheimer's Disease Repository Without Borders (ARWIBO), and ADNI. All preprocessed brain images were selected. The GARD consists of 81 AD subjects (39 males, 42 females; age ± SD = 71.86 ± 7.09 years, education level = 7.34 ± 4.88, range = 0–18), 171 cognitively normal HC subjects (83 males, 88 females; age ± SD = 71.66 ± 5.43 years, education level = 9.16 ± 5.54, range = 0–22), 39 patients with mAD (25 males, 14 females; age ± SD = 73.23 ± 7.09 years, education level = 8.20 ± 5.19, range = 0–18), and 35 patients with aAD (15 males, 20 females; age ± SD = 72.74 ± 4.82 years, education level = 7.88 ± 6.30, range = 0–18). The NACC includes 26 AD subjects (11 males, 15 females; age ± SD = 73.33 ± 9.43 years, education level = 14.44 ± 3.58, range = 0–18), 42 cognitively normal HC subjects (22 males, 20 females; age ± SD = 65.98 ± 11.91 years, education level = 15.89 ± 2.96, range = 0–22), 30 patients with mAD (10 males, 20 females; age ± SD = 75.52 ± 8.62 years, education level = 14.91 ± 3.45, range = 0–18), and 33 patients with aAD (16 males, 17 females; age ± SD = 73.12 ± 8.92 years, education level = 14.39 ± 4.08, range = 0–18). The ARWIBO consists of 29 AD subjects (10 males, 19 females; age ± SD = 71.2 ± 4.14 years, education level = 8.37 ± 9.31, range = 0–18), 33 cognitively normal HC subjects (16 males, 17 females; age ± SD = 65.5 ± 9.09 years, education level = 10.0 ± 6.82, range = 0–22), 34 patients with mAD (14 males, 20 females; age ± SD = 69.7 ± 7.11 years, education level = 7.67 ± 4.21, range = 0–18), and 25 patients with aAD (10 males, 15 females; age ± SD = 69.45 ± 3.22 years, education level = 7.97 ± 5.21, range = 0–18). The ADNI consists of 32 AD subjects (17 males, 15 females; age ± SD = 72.14 ± 4.21 years, education level = 9.41 ± 3.78, range = 0–18), 28 cognitively normal HC subjects (18 males, 10 females; age ± SD = 64.02 ± 6.45 years, education level = 11.41 ± 6.56, range = 0–22), 25 patients with mAD (12 males, 13 females; age ± SD = 69.14 ± 8.35 years, education level = 7.99 ± 4.20, range = 0–18), and 38 patients with aAD (22 males, 16 females; age ± SD = 67.11 ± 5.81 years, education level = 8.02 ± 7.10, range = 0–18).

Tables 1–4 demonstrate the demographics of the 326 subjects from the GARD, 121 subjects from the ARWIBO, 131 subjects from the NACC, and 123 subjects from the ADNI for this study. The clinical variables and distinguishing statistics in demographics among the research groups were determined using the Welch independent samples *t*-test. In this research, the significance level was 0.05, which is a normal alpha value. In the GARD data case, the rate for females was greater than that of other groups except for the EMCI group. The levels of education were completely disparate in the pairwise comparisons among study groups. According to the comparison among the groups, the AD groups had the lowest level of education. In this study, to gain unbiased estimated performance, every dataset was randomly split into two parts with a 70 : 30 ratio for training and testing. The approach involved training with a training algorithm code. We tested the remaining dataset using the trained algorithm. Moreover, the analysis of the group performance was classified in terms of accuracy, specificity, sensitivity, precision, and F1 score utilizing a unique test set.

### 2.2. MRI Acquisition

A brain image occupies space in three-dimensional (3D) images, so we could use volume data to fill this space. The volume data are measured voxels, which look like the pixels utilized to display images only in 3D.

Standard 3T T1-weighted images were obtained utilizing the volumetric 3D MPRAGE protocol with a resolution 1 × 1 × 1 mm (voxel size). All images were N4 bias corrected.

### 2.3. Feature Selection

Segmented MRI brain images have been used mostly for classification with machine learning and the subfield of machine-learning techniques. According to many types of studies, the subcortical part of the brain is easily affected by dementia and AD compared to the cortical part, but cortical thickness is an outstanding candidate for the treatment of AD. In this research, subcortical/cortical features were extracted by using MALPEM, and 138 features were achieved from 3D sMRI T1-weighted images. MALPEM is a collection of tools for distinguishing and visualization of cortical/subcortical parts of the brain based on the sagittal, axial, and coronal views in Figure 1. MALPEM was constructed using an automatic workflow consisting of several standard image-processing techniques, dividing 138 ROIs. In recent years, multiatlas segmentation has developed into one of the most accurate methods for the segmentation of T1-weighted images, mostly focusing on graph-cut or EM optimization. MALPEM [24] was evaluated as a top 3 method in a Grand Challenge on whole-brain segmentation at MICCAI 2012 (http://www.christianledig.com). The sMR images of all 701 subjects were segmented individually utilizing MALPEM as designated in previous research [3]. It consumed between 8 and 10 h for each subject. For this segmentation, the automatically explained neuromorphometrics brain atlas (*n* = 30; provided by Neuromorphometrics, Inc., under academic subscription, http://neuromorphometric/, last accessed 15 March 2018) was used. This atlas automatically distinguishes the whole-brain images into 40 noncortical and 98 cortical parts. MALP was utilized to acquire the specific probability of a brain atlas for sMRI brain images as *K,* which should be segmented [3]. This probability is integrated into the EM framework as a spatial anatomical task. *n* is indicated as a voxel of *K* by *j* = 1,…*n*; therefore, the intensities of the voxel *Z*_*i*_ ∈ *D*; image should be described as *K*={*Z*_1_,  *Z*_2_ … *Z*_*n*_}. The probabilistic priors are produced through the transformation of manually generated *L* atlases into the coordinate space of the unseen image. For the propagation of the tag, the *L* transformations were measured using a nonrigid registering technique based on free-form deformation, which follows a previous rigid technique and some alignment. By using a locally weighted multiatlas fusion strategy, the probabilistic atlas was designed for image intensity normalization and rescaling by the Gaussian weighted sum of squared differentiation. The estimated hidden segmentation employing the observed intensities *j* followed the approach of Van Leemput et al. [25]. It was considered that the observed log-transformed intensities of the voxels refer to a spatial class *N* and are dispensed with mean *φ*_*N* _ and standard deviation *ρ*_*N*_:

(1) $$\begin{array}{c} \psi \;=\;\left\{\left(\varphi_{1},\rho_{1}\right),\;\left(\varphi_{2},\rho_{2}\right),\ldots \ldots ,\left(\varphi_{N},\rho_{N}\right)\right\}. \end{array}$$

The global Markov random fields approach was used for applying the regularization of the resulting segmentation. The EM algorithm makes segmentations with very low-intensity variance within the region (intraclass variance) compared to the “gold-standard” segmentations. Therefore, normalized intraclass variance was determined for each region (*ρ*_*N*Gold,*k*_)  by averaging the normalized standard deviations (*ρN* /*φN*) of every group over the training subjects. Moreover, the averaged (averaged over all training subjects segmented with a leave-one-out strategy) distributed standard deviation was measured within every region assembled by the EM algorithm (*ρ*_EM,*k*_). By determining  Δ_*N*_ = (*p*_*N*Gold,*k*_ −  *p*_EM,*k*_)^2^, it was evaluated by which value the intraclass variance of the spatial group might be enhanced on average to match the gold-standard innates better [26]. The final segmentation was created by fusing the refined labels for this subset with the labels from the MALP approach for enduring parts. After completion of segmentation, all the segmented data were normalized to zero mean and component variance for every feature, as demonstrated in Figure 2, utilizing the ordinary scalar function of the scikit-learn library. According to normalization, *ξ* is a given data matrix where the subjects are in rows, and the features of subjects are in columns. The elements of normalized matrix illustrate *ξ* (*m, n*), and the equation is given by

(2) $$\begin{array}{c} {\xi \;}_{\text{norm},\left(m,n\right)}=\frac{{\xi \;}_{\left(m,n\right)}-\text{mean}\left({\xi \;}_{n}\right)}{\text{std}\left({\xi \;}_{n}\right)}. \end{array}$$

Then, for reduction of dimensionality, PCA was executed [27], with all features designed into a lower-dimensional space. PCA map features in a new *N*-dimensional subspace should be less than those in the initial *L*-dimensional space. The new *N* variance is the principal component, and every principal component eliminates the maximum variance that is accounted for in all accomplishing components. The principal components can be illustrated by the following equation:

(3) $$\begin{array}{c} {\text{PC}}_{j}=m_{1}k_{1}+m_{2}k_{2}+\cdots \cdots +m_{z}k_{z}, \end{array}$$

where PC_*j*_ is a principal component in *j*, *y*_*z*_ is an original feature in *z,* and *m*_*z*_ is a numerical coefficient of *y*_*z*_. The observed original features are greater than or equal to the number of principal components. The achieved principal components for AD versus HC are illustrated in Figure 3. The component number was regulated by controlling the features greater than 96%. The first principal component gained 96% among all the other 83 features received after passing all 138 features. Hence, the first component was utilized for the classification of EMCI versus LMCI as well.

### 2.4. Classification Method

Previously, the cortical and subcortical region features were extracted by using an automatic toolbox (MALP-EM) based on sMRI T1-weighted images. The feature vectors covering mean-centered voxel intensities were constructed by fusing all features. The classification method used here is designed to fuse two resources of features: subcortical volume and cortical thickness. The above features are utilized for a framework decision to distinguish AD from other subjects. Moreover, when comparing the classification for two-part brain images—cortical and subcortical—by RBF-SVM machine-learning classifiers, in some dataset cases, the cortical thickness was determined with good accuracy; in another case, the subcortical provided better results.

### 2.5. SVM

This machine-learning classifier is being used widely to investigate sMRI data [5, 12, 20]. RBF-SVM is suitable for binary classification for separable and nonseparable data. In the past decade, it has been employed as the most popular machine-learning tool in neuroimaging and neuroscience. This approach depends on selecting a critical point for the classification work. Support vectors are elements that are distinguished into two groups. RBF-SVM is a supervised learning classification algorithm and determines the optimal hyperplane that discriminates both modules with an extreme margin from support vectors during the training phase. The estimated hyperplane determines the classifier for the testing of a new data point. In some cases, such as linear ones, SVM might not guarantee a good result, so linear SVM is expanded by utilizing a kernel trick. The central idea of kernel methods is that the input data are designed into a higher-dimensional plane employing linear and nonlinear functions for known kernels. SVM kernels exploit nonlinear and linear RBF. Moreover, the linear kernel is a superior case of RBF. The linear kernel with a penalty parameter *Ĉ* has the same presentation as the RBF kernel with the parameters (*c*, *y*). The RBF has two parameters, *c* and *y,* that are good for an assumed problem. The main goal of analyzing good (*c*, *y*) is to enable the classification method to predict testing data accurately.

## 3. Results and Discussion

### 3.1. Background

In this experiment, the proposed method utilized the RBF-SVM classification algorithm. Then, all extracted features were split into the cortical thickness and subcortical volume in the MALPEM toolbox to distinguish between the AD versus HC and EMCI versus LMCI groups. This classification was performed to recognize how well the approach performs on the sMRI 3D images. In the beginning stage, normalization was designed for every subject. Furthermore, the PCA reduction of dimensionality method was employed to select the optimal number of principal components for every binary classification. In a different binary classification group, different numbers of principal components were gained. Moreover, to confirm the robustness of the classification result, 10-fold stratified K-fold (SKF) cross-validation (CV) was utilized.

### 3.2. Evaluation

The set of subjects was randomly split into two groups in a 70 : 30 ratio for training and testing to obtain unbiased estimates of the performance. The training set was used for analyzing the optimal hyperparameters of every technique and classifier. Furthermore, the testing set was utilized for classification achievement. For optimal hyperparameter estimation, SKF-CV was used based on the training set. Following the LIBSVM library, the linear SVM *Ĉ* kernel value and *c, y* parameters of the kernel were regulated. While choosing the default parameter features, SVM performed poorly on the preliminary data. Hence, to regulate the optimal parameters for *c* and *y*, the grid search method was used before *c* and *y* were utilized for training. For *c* and *y*, CV accuracy was selected as the best parameter. In this work, two parameters were set—*c* = 1 to 10 and *y* = (1*e*^−4^, 1*e*^−2^, 0.0001)—for every classification group. Then, to analyze the classifier for the training groups, the obtained optimized values were regulated. The assessment of binary classifiers was determined by using confusion metrics, which is a precise test covering binary classification tasks. The diagonal elements of the metric demonstrate the corrected predictions created by the classifier. Then, elements could be split into two groups that express the controls of correctly identified true positive (TP) and true negative (TN). However, the subjects classified incorrectly can be defined as false positive (FP) and false negative (FN). The determination of accuracy in equation (4) is the number of samples in which the classifiers regulated correctly.

(4) $$\begin{array}{c} \text{Acc}=\frac{\text{TP}+\text{TN}}{\text{TP}+\text{TN}+\text{FP}+\text{FN}}. \end{array}$$

Moreover, considering only accurate measurement was not sufficient for the unstable class dataset and resulted in misleading estimation. Hence, the additional four assessment metrics should be adjusted: sensitivity, specificity, precision, and F1 score. They are designated as follows:

(5) $$\begin{array}{c} \text{Sen}=\frac{\text{TP}}{\text{TP}+\text{FN}}, \end{array}$$

(6) $$\begin{array}{c} \text{Spec}=\frac{\text{TN}}{\text{TN}+\text{FP}}, \end{array}$$

(7) $$\begin{array}{c} \text{Ppv}=\frac{\text{TP}}{\text{TP}+\text{FP}}. \end{array}$$

(8) $$\begin{array}{c} \text{F}1\text{ score}=\frac{2\text{TP}}{2\text{TP}+\text{FP}+\text{FN}}. \end{array}$$

Sensitivity, given in equation (5), illustrates the accuracy of the predicted group. Specificity, given in equation (6), illustrates the accuracy of the predicted absence group. Sensitivity, which is also called “recall” or “probability of detection,” is the proportion of actual positives that are correctly determined. Similarly, specificity investigates the proportion of actual negatives that is not included in the class. Precision, given in equation (7) (positive predictive value), is the element of appropriate incidences between the repossessed incidences. F1 score, given in equation (8), determines the accuracy of a test. To assess that each method performs significantly better than a random classifier, the Cohen kappa and Jaccard distance were utilized. Cohen kappa determination is usually utilized to analyze interrater reliability. Rater reliability demonstrates the degree to which the data represented in the research are appropriate illustrations of the variables evaluated. The Cohen [28] is a statistic helpful for an interrater accuracy testing. The determination of the Cohen kappa can be executed based on the following equation:

(9) $$\begin{array}{c} \text{k}=\frac{\mathrm{Pr}\left(a\right)-\text{Pr}\left(e\right)}{1-\text{Pr}\left(e\right)}. \end{array}$$

Here, *P*_*r*_ (*a*) demonstrates the observed agreement and *P*_*r*_ (*e*) illustrates chance agreement. The kappa can range between −1 and + 1, and the kappa result is explained as follows: if the values are ≤0, there is no agreement; between 0.01 and 0.20, there is minor arrangement; between 0.21 and 0.40, there is known fair agreement; between 0.41 and 0.60, there is moderate agreement, between 0.61 and 0.80, there is substantial agreement; and from 0.81 to 1.00, there is nearly perfect agreement [29]. The Jaccard index determines how close the commonality of the two datasets can be a measured [30]. The Jaccard coefficient is given in the following equation:

(10) $$\begin{array}{c} J\left(M,N\right)=\frac{\left|M\cap^{}N\right|}{\left|M\cup^{}N\right|}. \end{array}$$

The Jaccard index is a statistic utilized for measuring the diversity and similarity of sample sets.

The range of Jaccard coefficient measures from 0% to 100% is as follows:

Jaccard index = (the amount in equal sets)/(the amount in either set) × 100.

The process of calculating the Jaccard index is as follows: (1) calculate the number of both members that are proportional for both sets, (2) calculate the entire number of members (proportional and nonproportional), and split the number of common members (1) by the entire number of members (2), and (3) multiply by 100 [31].

### 3.3. Classification Results

The binary classification was utilized to analyze subcortical volume and cortical thickness volume of AD versus HC and EMCI versus LMCI subject groups. The results of classification are demonstrated in Table 5, and all results are illustrated in Figures 4(a) and 4(b). Kappa and Jaccard are shown in Figures 4(c) and 4(d). All processes were performed in a 64-bit Python 3.6 environment on Intel Core i7-8700 at 3.20 Hz and 16 GB of RAM running Ubuntu 16.04.

#### 3.3.1. Binary Classification: AD versus HC and EMCI versus LMCI

According to the four datasets, two binary groups—AD versus HC and EMCI versus LMCI—were classified with subcortical volume and cortical thickness features by utilizing the RBF-SVM classification algorithm, and the result is illustrated in Table 5.

*(1). AD versus HC.* The result of classification for AD versus HC is given in Table 5 and Figures 4(a) and 4(c). In every classification situation, the database was divided into two separations in a 70 : 30 ratio. Each dataset shows better results for kappa and Jaccard statistics in the RBF-SVM classification technique. In the kappa statistics case, the GARD dataset cortical thickness feature gives the highest interrater reliability of 0.9342, and the ARWIBO dataset subcortical volume feature has 0.8939. In the Jaccard statistics case, the GARD dataset cortical thickness is 0.9091, the highest, and the ARWIBO dataset subcortical volume feature is 0.8889. Moreover, the GARD cortical thickness has a good F1 score, precision, specificity, and sensitivity (98.18%, 96.87%, 95.24%, and 98.18%, respectively).

*(2). EMCI versus LMCI.* The classification performance for EMCI versus LMCI is shown in Table 5 and Figures 4(b) and 4(d). Similarly, the kappa statistics for the GARD dataset subcortical volume feature shows the highest result—0.9043—and the ARWIBO dataset cortical feature is 0.8979. The Jaccard statistic for the GARD dataset subcortical volume feature had the highest result—0.9186. The NACC dataset subcortical volume feature is 0.9167. Furthermore, the GARD dataset subcortical volume feature has better results, with an F1 score, precision, specificity, and sensitivity of 96.45%, 100%, 100%, and 92.75%, respectively, compared to the cortical thickness.

#### 3.3.2. Comparison with Related Recently Published Methods

As mentioned above, in the proposed method, four datasets were used: GARD, NACC, ARWIBO, and ADNI. Except for the GARD dataset, all are available for the public, and anyone can download them. The websites available are NACC (https://www.alz.washington.edu/), ARWIBO (https://www.gaaindata.org/partner/ARWIBO), and ADNI (http://adni.loni.usc.edu/).

There are 701 subjects: 326 (GARD), 131 (NACC), 121 (ARWIBO), and 123 (ADNI). The ages of all subjects are more than 47, and converting of mild cognitive stage to AD between 0 and 18 months. For segmentation, the T1-weighted sMRI imaging modality was utilized from each dataset. Moreover, the results of the proposed method were compared to recently published results, as shown in Tables 6 and 7.

Tripathi et al. [13] proposed a method that used the RBF and linear SVM classifier for the automated pipeline which distinguishes subjects between AD, LMCI, EMCI, and HC with subcortical and hippocampal features gained from spherical harmonics (SPHARM-PDM) process by utilizing the ADNI dataset. The combination of voxel and SPHARM features shows 88.75% accuracy, 83.10% sensitivity, and 91.58% specificity for an AD versus HC group with a linear kernel SVM, whereas, for EMCI versus LMCI group, the same combined features show 70.95% accuracy, 75.56% sensitivity, and 65.47% specificity with linear SVM. Likewise, another study by Zhang et al. [19] used an SVM with nested cross-validation to distinguish the features into two groups to gain balanced results. The slow-5 frequency band shows 83.87% accuracy, 86.21% sensitivity, and 81.82% specificity for EMCI versus LMCI cohort by using the ADNI dataset. Gorji and Naima [17] have utilized CNN deep learning algorithms in their pipeline and utilizing it they have obtained a 93% accuracy, 91.48% sensitivity, and 94.82% specificity for EMCI versus LMCI using sagittal features from an MRI image. Furthermore, Nozadi and Kadoury [15] compared the FDG and AV-45 biomarkers of PET image and then employed RBF-SVM and RF for distinguishing AD, NC, EMCI, and LMCI with six groups by using ADNI dataset. Their approach showed accuracies of 91.7% and 91.2% for AD versus NC, each of RBF-SVM and RF with FDG-PET image modality. On the other hand, AV45 illustrates accuracies of 90.8% and 87.9% for AD versus NC with RBF-SVM and RF. For EMCI versus LMCI, FDG-PET provides better 53.9%, 64.1% accuracies compared with AV45 results in RBF-SVM and RF classifier. Gupta et al. [5] proposed a method utilizing the GARD dataset as a known private dataset, and the OASIS dataset was used for comparison. The four classifiers were utilized for binary and tertiary classification and achieved better results according to the classifier. For AD versus HC, the softmax classifier showed the highest accuracy of 99.34%, 100% specificity, and a precision of 100%. For the HC versus mAD case, the SVM classifier had an accuracy of 99.2% and a specificity and precision of 100%. The mAD versus aAD SVM provided good results as well, such as a 97.77% accuracy, 100% sensitivity, and 97.95% F1 score. In tertiary classification, SVM had the best accuracy of 99.42%, 99.18% sensitivity, and 99.99% precision in AD versus HC versus mAD. In AD versus HC versus aAD, the NB classifier had 96.53% accuracy, 95.88% sensitivity, and 97.64% specificity.

## 4. Discussion

In this research, the RBF-SVM method was employed for classification of subjects with AD versus HC and EMCI versus LMCI based on anatomical T1-weighted sMRI. The proposed method is shown in Figure 3. The subjects were divided into a ratio of 70 : 30 for training and testing purposes before being passed to the classifier. Then, the dimensionality reduction method was utilized by using the PCA function from the scikit-learn library. Subsequently, for the SVM classifier, the optimal structure value was regulated by employing SKF-CV and a grid search. Then, the above features were utilized to instruct the SVM classifier using the training dataset, and the testing dataset was assessed using the training method to determine the performance. The proposed method shows more than 90% accuracy for all datasets based on cortical and subcortical features in the AD versus HC groups. In the GARD dataset case, cortical thickness had the best accuracy, 97.37%, a sensitivity of 98.18%, and an F1 score of 98.18%. Moreover, kappa and Jaccard statistical analyses resulted in more than 0.80 for all datasets in AD versus HC binary classification.

In the EMCI versus LMCI group, GARD subcortical volumes had the highest accuracy among all datasets—95.45% accuracy, 100% precision, and 100% specificity. The Cohen kappa and Jaccard statistical volume produced good results as well. Moreover, GARD had a good AUC for the subcortical volume and cortical thickness of both groups, as given in Figure 5. In the ADNI dataset case (AD versus HC), the cortical thickness showed 100% specificity, 100% precision, and an accuracy of 91.57%. The EMCI versus LMCI subcortical volume had a specificity and precision of 100%. In the ARWIBO dataset case (AD versus HC), the subcortical volume had 100% sensitivity, 94.74% accuracy, and 95.24% F1 score, but for EMCI versus LMCI, the cortical thickness had a specificity of 100%, precision of 95.66%, and 94.74% F1 score. Furthermore, in the NACC dataset case (AD versus HC), the subcortical volume was 100%, with 100% specificity and precision and a 96.55% F1 score. Likewise, the EMCI versus LMCI subcortical volume had a specificity and precision of 100% and an accuracy of 94.74%. In both binary classifications, the proposed method obtained good results compared to those proposed in other works. In addition, the Cohen kappa and Jaccard results demonstrate excellent statistical analysis for ADNI, GARD, ARWIBO, and NACC.

## 5. Conclusions

A novel method for automatic classification, AD from MCI (early or late converted to AD) and an HC, was developed by utilizing the features of cortical thickness and subcortical volumes. The features were extracted from a MALPEM toolbox, and classification was performed by the RBF-SVM classifier based on the GARD dataset. They were compared to three datasets. The results of this research prove that the proposed approach is efficient for future clinical prediction between the subcortical view of EMCI versus LMCI and the cortical view of AD versus HC, which are shown in Table 5. Based on the subcortical volume and cortical thickness, the proposed method obtained different accuracies according to the different databases, such as the GARD and NACC dataset AD versus HC group cortical thickness accuracies of 97.37% and 95.24%. The subcortical volumes of ARWIBO and NACC for the AD versus HC group were 94.74% and 94.56%.

In this research, only the subcortical volume and cortical thickness features were considered for the classification procedure. In the future, it is planned to examine classifier multimodality features of the brain biomarkers and nonimaging biomarkers for diagnosis of AD. Furthermore, we are planning a future work to compare state-of-the-art and recently published methods with different available datasets for early prediction of AD.

## Figures and Tables

**Figure 1:** Cross-sectional segmentation results for T1-weighted MRI images: (a) axial, (b) coronal and sagittal, and (c) view planes.

**Figure 2:** Proposed technique workflow.

**Figure 3:** Number of principal components for AD versus HC.

**Figure 4:** Classification reports of four datasets—ADNI-C (cortical), ADNI-S (subcortical), ARWIBO-C (cortical), ARWIBO-S (subcortical), NRCD-C (cortical), NRCD-S (subcortical), NACC-C (cortical), and NACC-S (subcortical)—with measurement performance (AUC, accuracy, sensitivity, specificity, precision, and F1 score): (a) AD versus HC, (b) EMCI versus LMCI, classification reports of four datasets with measurements of kappa and Jaccard, (c) AD versus HC, and (d) EMCI versus LMCI.

**Figure 5:** AUC-ROC performance for the GARD dataset: (a) AD versus HC cortical thickness, (b) AD versus HC subcortical, (c) EMCI versus LMCI cortical, and (d) EMCI versus LMCI subcortical.

**Table 1:** Demographic characteristics of the studied population (from the GARD database).

Group	Subject number	Age	Gender		Education
			M	F	
AD	81	71.86 ± 7.09 [56–83]	39	42	7.34 ± 4.88 [0–18]
EMCI	39	73.23 ± 7.34 [49–87]	25	14	8.20 ± 5.19 [0–18]
LMCI	35	72.74 ± 4.82 [61–83]	15	20	7.88 ± 6.30 [0–18]
HC	171	71.66 ± 5.43 [60–85]	83	88	9.16 ± 5.54 [0–22]

**Table 2:** Demographic characteristics of studied population (from the ARWIBO dataset).

Group	Subject number	Age	Gender		Education
			M	F	
AD	29	71.24 ± 14.09 [59–80]	10	19	8.37 ± 3.78 [0–18]
EMCI	34	69.7 ± 7.11 [51–82]	14	20	7.67 ± 4.21 [0–18]
LMCI	25	69.45 ± 3.22 [59–79]	10	15	7.97 ± 5.21 [0–18]
HC	33	65.59 ± 9.12 [58–83]	16	17	10.06 ± 3.43 [0–22]

**Table 3:** Demographic characteristics of studied population (from the NACC dataset).

Group	Subject number	Age	Gender		Education
			M	F	
AD	26	73.33 ± 9.43 [50–78]	11	15	14.44 ± 3.58 [0–18]
EMCI	30	75.52 ± 8.62 [47–85]	10	20	14.91 ± 3.45 [0–18]
LMCI	33	73.12 ± 8.92 [58–80]	16	17	14.39 ± 4.08 [0–18]
HC	42	65.98 ± 11.91 [59–83]	22	20	15.89 ± 2.96 [0–22]

**Table 4:** Demographic characteristics of studied population (from the ADNI dataset).

Group	Subjects number	Age	Gender		Education
			M	F	
AD	32	72.14 ± 4.21 [54–79]	17	15	9.41 ± 3.78 [0–18]
EMCI	25	69.14 ± 8.35 [48–83]	12	13	7.99 ± 4.20 [0–18]
LMCI	38	67.11 ± 5.81 [60–81]	22	16	8.02 ± 7.10 [0–18]
HC	28	64.02 ± 6.45 [63–84]	18	10	11.41 ± 6.56 [0–22]

**Table 5:** Result of four datasets for the subcortical and cortical parts for AD versus HC and EMCI versus LMCI.

AD vs. HC	Classifier	AUC	ACC	SEN	SPEC	PRE	F1	Kappa	Jaccard
ADNI cortical	SVM-RBF	91.67	91.57	81.82	100	100	90	0.8108	0.8333
ADNI subcortical		90.45	90.48	90.91	90	90.91	90.91	0.8091	0.8182
ARWIBO cortical		89.44	89.47	90	88.89	90	90	0.7889	0.8
ARWIBO subcortical		95.45	94.74	100	88.89	90.91	95.24	0.8939	0.8889
NRCD cortical		97.5	97.37	98.18	95.24	96.87	98.18	0.9342	0.9091
NRCD subcortical		95.71	93.42	96.3	86.36	94.55	95.41	0.8379	0.7917
NACC cortical		96.88	95.24	100	83.33	93.75	96.77	0.8772	0.8333
NACC subcortical		92.86	94.56	93.33	100	100	96.55	0.8889	0.8571
EMCI vs. LMCI	Classifier	AUC	ACC	SEN	SPEC	PRE	F1	Kappa	Jaccard
ADNI cortical	SVM-RBF	81.75	81.25	75	87.5	85.71	80	0.725	0.7158
ADNI subcortical		88.89	87.5	77.78	100	100	87.5	0.7538	0.7778
ARWIBO cortical		94.44	93.24	90	100	95.66	94.74	0.8979	0.8889
ARWIBO subcortical		95	94.87	88.89	92.75	100	94.12	0.8889	0.9012
NRCD cortical		92.86	90.91	91.45	100	100	88.89	0.8136	0.8271
NRCD subcortical		96.43	95.45	92.75	100	100	96.45	0.9043	0.9186
NACC cortical		91.67	89.47	87.78	89.57	90.24	87.5	0.7989	0.8133
NACC subcortical		95.83	94.74	92.56	100	100	93.33	0.8902	0.9167

**Table 6:** Comparison of recently published works.

AD vs. HC						
Years	Approach	Dataset	ACC	SEN	SPEC	Classifier
**2017**	Tripathi et al. [13]	ADNI	85.98	75.55	90.30	RBF-SVM
**2018**	Nozadi and Kadoury [15]	ADNI	89.3	88.8	85.9	RBF-SVM
**2018**	Gupta et al. [5]	NRCD	99.34	98.14	100	Softmax
		OASIS	98.40	93.75	100	
**2019**	Proposed method	NRCD	**97.37**	**98.18**	**95.24**	RBF-SVM
		NACC	95.24	100	83.33	
		ARWIBO	94.74	100	88.89	
		ADNI	91.57	81.82	100	

**Table 7:** Comparison of recently published works.

EMCI vs. LMCI						
Years	Approach	Dataset	ACC	SEN	SPEC	Classifier
**2017**	Tripathi et al. [13]	ADNI	70.29	73.95	66.01	RBF-SVM
**2018**	Nozadi and Kadoury [15]	ADNI	67.6	70.1	70.7	RBF-SVM
**2018**	Gupta et al. [5]	NRCD	95.55	100	90.9	Softmax
**2019**	Zhang et al. [19]	ADNI	83.87	86.21	81.82	RBF-SVM
**2019**	Gorji and Naima [17]	ADNI	93.00	91.48	94.82	CNN
**2019**	Proposed method	NRCD	**95.45**	**92.75**	**100**	RBF-SVM
		NACC	94.74	92.56	100	
		ARWIBO	94.87	88.89	92.75	
		ADNI	87.50	77.78	100	

## Data Availability

The Gwangju Alzheimer's disease and Related Dementia (GARD) dataset was used to support the findings of this study. The GARD is a private dataset that was generated in Chosun University hospitals, and it belongs to Chosun University. The authors cannot share it or make it available online for privacy reasons. Moreover, to compare the proposed approach with other datasets, the authors downloaded the NACC dataset from https://www.alz.washington.edu, the ARWIBO one from https://www.gaaindata.org, and the ADNI one from http://adni.loni.usc.edu.
